# IoT-Based Smart Health Monitoring System for COVID-19 Patients

**DOI:** 10.1155/2021/8591036

**Published:** 2021-11-16

**Authors:** Mohammad Monirujjaman Khan, Safia Mehnaz, Antu Shaha, Mohammed Nayem, Sami Bourouis

**Affiliations:** ^1^Department of Electrical and Computer Engineering, North South University, Bashundhara, Dhaka 1229, Bangladesh; ^2^Department of Information Technology, College of Computers and Information Technology, Taif University, P.O. Box 11099, Taif 21944, Saudi Arabia

## Abstract

During the ongoing COVID-19 pandemic, Internet of Things- (IoT-) based health monitoring systems are potentially immensely beneficial for COVID-19 patients. This study presents an IoT-based system that is a real-time health monitoring system utilizing the measured values of body temperature, pulse rate, and oxygen saturation of the patients, which are the most important measurements required for critical care. This system has a liquid crystal display (LCD) that shows the measured temperature, pulse rate, and oxygen saturation level and can be easily synchronized with a mobile application for instant access. The proposed IoT-based method uses an Arduino Uno-based system, and it was tested and verified for five human test subjects. The results obtained from the system were promising: the data acquired from the system are stored very quickly. The results obtained from the system were found to be accurate when compared to other commercially available devices. IoT-based tools may potentially be valuable during the COVID-19 pandemic for saving people's lives.

## 1. Introduction

Currently, the COVID-19 pandemic is one of the major global issues faced by health organizations. As of November 19, 2020, the total number of people worldwide confirmed to have been infected with SARS-COV-2 is more than 56.4 million, while the total number of fatalities from the coronavirus is more than 1.35 million, thereby proving that COVID-19 cases are surging worldwide [1].

In Bangladesh, presently, there are a total of 445,281 positive COVID-19 cases, while the coronavirus fatality toll is 6350 as of November 21, 2020 [2]. COVID-19 patients have several symptoms, such as fever, shortness of breath, decrease in oxygen saturation level, dry cough, diarrhea, vomiting, sore throat, headache, loss of taste and smell, body pain, and abnormal pulse rate [3]. Among these symptoms, high fever, low oxygen saturation level, and abnormal pulse rate are considered serious. Low oxygen saturation level and shortness of breath cause hypoxemia and hypoxia, respectively. Patients who suffer from hypoxemia and problems with pulse rate have a less chance of survival. Sometimes, patients do not recognize hypoxemia and an increasing rate of pulse, and they subsequently die without receiving proper treatment. Therefore, it is important for COVID-19 patients to be regularly informed about their health conditions, especially body temperature, heart rate, and oxygen saturation (SpO2) [4, 5].

As a person enters old age, it becomes increasingly vital for them to undergo standard medical health checkups. Since it may be time-consuming and difficult for most people to get regular health checkup appointments, IoT-based arrangements can be beneficial to individuals for routine health checkups [4, 5]. IoT technology has developed into an imperative innovation with applications in numerous areas. Specifically, it refers to any system of physical devices that obtain and exchange information over wireless systems without human mediation [6, 7]. With a significantly large increase in active COVID-19cases during the second wave, every country (including Bangladesh) faces issues in providing proper treatment to their patients. Pulse rate and body temperature are the most basic markers of human health. The pulse rate, also known as the beat rate, is the number of pulses per minute. The normal pulse rate ranges between 60 and 100 beats per minute for typical individuals. The average resting pulse rate for adult males and females is approximately 70 and 75 bpm, respectively [8, 9]. Females over the age of 12 typically have higher pulse rates than men. However, the pulse rate for COVID-19 patients is abnormal and requires aid from an emergency medical assistant. The internal heat level of an individual depends on various factors, such as surrounding temperature, gender, and dietary pattern, and the temperature ranges between 97.8°F (36.5°C) and 99°F (37.2°C) in healthy adults [9–11]. Various factors, such as influenza, low-temperature hypothermia, and other diseases, may prompt a fluctuation in body temperature. In most diseases, including COVID-19, fever is a common symptom; therefore, it is essential to regularly measure the body temperature. Oxygen saturation is also an important factor inCOVID-19patients. The normal oxygen saturation (SpO2) of the human body ranges from 95 to 100%. If the SpO2 (oxygen saturation) level of a COVID-19 patient is below 95%, they require emergency medical care. SARS-COV-2 coronavirus produces silent hypoxia, that is, SpO2 < 90%without shortness of breath. Silent hypoxia can be diagnosed by monitoring SpO2 using a pulse oximeter [10, 11]. If the oxygen saturation level of a COVID-19 patient is significantly low, the patient may die. To manage COVID-19, it is crucial to monitor early symptoms such as fever, cough, heart rate, and SpO2.

Recently, different types of devices have been used to measure these values. For example, a fingertip pulse oximeter, which is used to measure SpO2 and pulse rate, is commercially available in most countries [12]. The deluxe handheld pulse oximeter is also commercially available, which can measure SpO2 and heart rate; although, it is priced at approximately 299 USD [13]. A wrist-worn pulse oximeter is available across the counter and can be used to measure SpO2 and heart rate. This device, like the abovementioned devices, does not include body temperature measurement features. The wrist-worn pulse oximeter costs 179 USD, rendering it expensive. Analog and digital thermometers are currently available in the market [14], but most of them are expensive [12]. The devices mentioned earlier are not based on IoT. Some of them show values, but it is cumbersome to obtain measurements from different devices. Therefore, in Bangladesh, it is difficult for a doctor to obtain updates from all patients at once. There is a demand for rapid monitoring of COVID-19 patients with serious symptoms. With the help of technology, it is possible for patients to receive COVID-19 treatment from home using their mobile phones [15]. This system helps patients with fever, low oxygen saturation, and an increasing or decreasing pulse rate. A person's pulse rate depends on their age, body size, heart health, and emotional stability [16]. The oxygen saturation and pulse rate are related because when a patient's oxygen level falls, their pulse rate increases. The IoT-based smart healthcare system is a real-time patient monitoring system, which has significantly aided the healthcare industry [17]. Recently, IoT-based smart healthcare devices have gained increased attention from a research perspective. The development of smart healthcare monitoring systems in an IoT environment is provided in the reviewed literature [18]. In this study, we used an Android-based pulse-monitoring system with a temperature sensor, a SpO2 sensor, and a heart rate sensor. In [19], the SpO2 measurement sensor was not used, and they shared the measured data on the internet. An IoT-based lung function monitoring system for asthma patients was proposed in [20], in which the temperature, SpO2, and pulse rate were not involved. Arduino, Android, and microcontroller-based heart rate monitoring systems have been proposed in [21, 22]. The system in [23] is based on the Arduino Uno and cloud computing, in which only a hardware prototype was produced. However, there are no real-world testing data available. In [24], a mobile application-based heart rate monitoring device was demonstrated. The patient's pulse rate was measured using a pulse rate sensor in this system, and the data were analyzed using Arduino. The measured information was delivered to the Android application. In the investigation, the number of sensors used was limited [24]. Different authors have presented different IoT-based wireless health-monitoring systems. However, presumably, IoT-based smart systems for measuring temperature, heart rate, and SpO2 for COVID-19 patients in one device have not been presented so far.

The main objective of this research is to develop and implement a novel IoT-based smart health monitoring system for COVID-19 patients based on human body temperature, pulse, and SpO2.The system can display measured human body temperature, oxygen saturation level, and pulse rate through a mobile application, which has been developed so that the patient can seek medical attention even if the specialist is physically unavailable. To treat a COVID-19 patient, a doctor requires the patient's oxygen saturation level and pulse rate. By using our proposed system, patients can inform doctors about their health conditions. This device can benefit COVID-19 patients as well as those suffering from other diseases, such as chronic obstructive pulmonary disease (COPD) and asthma. In 2005, COPD caused 5% of total deaths worldwide and could be a worldwide open health concern in the future [25]. Therefore, this system could be beneficial for such patients. If a patient's oxygen saturation and pulse rate is abnormal, the system immediately produces a buzz to alert the patient. Therefore, through a mobile application, patients can analyze the measured oxygen saturation level, pulse rate, and body temperature to avoid critical health conditions. This system was tested on five human test subjects. The patient and doctor can read the data throughout the day by using the mobile application. This system also has the ability to measure body temperature, which has not been included in any other research.

## 2. Material and Methods

### 2.1. Methods

A block diagram and flowchart were used as guides to visualize the arrangement of steps to be followed throughout the system management process. When the cycle stream was created, it directed essential periods of any future activities from the beginning to the end of a system. Circuit diagrams were utilized for the planning, development, and support of electrical and electronic gears. For a well-developed system, these diagrams were truly significant.  Figure 1 shows a block diagram of the proposed system. The system block diagram shows that when the power of the system is switched on, the sensor starts taking values. Here, the system has two types of sensors for measuring SpO2, pulse rate, and temperature. The sensors measure the physiological data from a human body and then pass the analog values to the Arduino, which converts them into digital data. The server sends the measured data to the mobile application and displays the data through an LCD display simultaneously. From the mobile application and device, users can monitor the temperature level, oxygen saturation (SpO2), and pulse rate.

Figure 2 shows the flow chart of the system. When the power of the device is activated, it starts measuring values and sends it to the main controller, Arduino Uno, and Node MCU. The Node MCU transmits the measured value to the fixed server. The system then displays measured temperature, pulse rate, and SpO2; if the measured oxygen saturation is below 95% and the pulse rate is less than 60 or greater than 90, the system sends an alert to both the doctor and the patient. Users can see the measured value through a mobile application, and simultaneously, users can see the value through the device's LCD display.

Figure 3 shows the block diagram of the whole circuit system. This diagram shows the pin connection between Arduino Uno, node MCU, Bluetooth module, SpO2 sensor, temperature sensor, and power supply of the system. This circuit diagram is designed using the Proteus Design Suite software. The active power button turns on the fully automated system. The sensors measure the data and send them to the processing unit, after which the data will be available on the mobile application as discussed earlier.

### 2.2. Hardware Materials Used

The system consists of two parts: the equipment and the mobile application. Both parts are fundamental to the system. The health monitoring system can measure oxygen saturation, pulse rate, and human body temperature. This multifunction system requires several components to be implemented. Implementation is achieved by performing activities portrayed in a work arrangement. For making the system successful, design implementation plays an important role. The components required to execute this system are briefly described below.  Table 1 lists the required hardware components, their quantities, and the cost of the products. The total cost of the hardware components for this system is 6120 Bangladeshi Taka, which is equivalent to 71.50 US dollars.

#### 2.2.1. Arduino Uno

There are several types of commercially available Arduino boards, such as Arduino Uno, Arduino Due, Arduino Mega, and Arduino Leonardo. The Arduino Uno has 20 I/O pins, 14 digital I/O pins, and six analog I/O pins. The Arduino Due has 54 digital I/O pins, 12 analog input pins, and two analog output pins. The Arduino Mega has 54 digital I/O pins, 16 analog inputs, and zero output pins. The Arduino Leonardo has 20 digital I/O pins, 12 analog inputs, and zero output pins [26]. To implement the system, we used the Arduino Uno because the pin configuration of this module fulfills the requirements of our system and is the main controller of the system. It is one of the most famous open-source microcontroller boards based on ATmega328p. This microcontroller is programmable using an Arduino IDE. In this system, it plays a crucial role and works as an interface between the sensors and the other IoT gadgets.  Figure 4 shows the model of the Arduino Uno.

#### 2.2.2. Pulse Sensor (MAX30100)

MAX30100 is a sensor that can measure blood oxygen saturation level and pulse rate.  Figure 5 shows the prototype of the SpO2 Pulse Sensor (MAX30100). Saturation of peripheral oxygen (SpO2) is a calculation of blood vessel oxygen saturation, which refers to the amount of oxygenated hemoglobin in the blood. In a human body, ordinary SpO2 values range from 90to 100%. In this system, a MAX 30100 pulse oximeter was suitable. It is a coordinated beat oximeter and heart rate sensor arrangement, which provides precise values. This sensor combines two LEDs, a photo detector, optimized optics, and low-noise analog flag handling to identify beat oximetry and heart rate signals; hence, it is suitable for this system.

#### 2.2.3. Bluetooth Module

There are many types of commercially available Bluetooth modules. We used the HC05 Bluetooth module for our system because it is user-friendly. The HC05 module is a type of Bluetooth serial port protocol module designed for wireless communication with Bluetooth-enabled devices and also communicates with microcontrollers using serial communication. This Bluetooth module has a range of 10 m and uses the 2.45-GHz frequency band. It has a data transfer rate of approximately1 Mbps. It can operate with a power supply of 4–6 V. The HC05 Bluetooth module has two operational modes: the command mode and the data mode [28].  Figure 6 shows the prototype of the HC05 Bluetooth module.

#### 2.2.4. Node MCU

We used the node MCU ESP8266 for this system, which is a wireless module, because the ESP8266 microcontroller has Wi-Fi capability, and the node MCU has a wireless system that can send data to a server. The node MCU has an asynchronous receiver-transmitter serial communication module, which enables it to communicate with the Bluetooth module. The node MCU ESP8266 microcontroller can operate with a power supply of 3.3 V operating voltage and a 7 to 12 V input voltage. It has a flash memory of 4 Mb and an SRAM of 64 Kb. It has 16 digital input and output pins and one analog input pin. The node MCU also has a PCB antenna [30]. The node MCU wireless module sends the measured pulse rate, oxygen saturation, and temperature to the server. This component was chosen because it links the server IP address to the node MCU to obtain the measured value through a mobile application. The node MCU is an open-source Lua-based firmware and an advancement board. It is specially designed for IoT-based applications, and this component plays a vital role in our system.  Figure 7 shows the prototype of the node MCU ESP8266 microcontroller.

#### 2.2.5. Buck Converter

The buck converter is a well-known and simple type of DC-DC converter. We used buck converters in our system because they produce an output voltage that is less than their input. This converter is utilized for proficient control transformation that amplifies battery life and decreases warmth.  Figure 8 shows the prototype of the buck converter.

#### 2.2.6. 16 × 2 LCD Display

A 16 × 2 liquid crystal display (LCD) is a well-known alphanumeric LCD display module, that is, it can show both letters and numbers. It has 16 columns and two rows which are useful in various systems. We used this display to show the measured pulse rate, oxygen saturation, and temperature. Here, each character is shown in a 5 × 8 pixel matrix. The operating voltage of the 16 × 2 LCD display is 4.7 to 5.3 V. Its current consumption is 1 mA when not illuminated by a backdrop [33].  Figure 9 shows the prototype of a 16 × 2 LCD display.

#### 2.2.7. DS18B20 Sensor

Figure 10 shows the DS18B20 sensor that works with the technique for 1-wire correspondence. It requires only the information pin related to the microcontroller with a draw-up resistor, and the other two pins are utilized to control. The pull-up resistor is used to keep the line in a high state when transport is not being operated. This sensor is used for the precise measurement of temperature. The temperature measured by the sensor will be absent in a 2-byte register inside the sensor. These data can be examined through the 1-wire procedure by sending them in an arrangement of data. There are two types of commands to be sent to examine the values: one could be a ROM command, and the other may be a working command [34].

### 2.3. Software Implementation

The mobile application was created by using Massachusetts Institute of Technology (MIT) App Inventor. MIT App Inventor is an online stage in which students can develop mobile applications. System designers can implement mobile applications for both iOS and Android using the MIT App Inventor. To implement the mobile application, a firebase is used as the backend server to store the data. Java and JavaScript are the languages used to develop this application [35].

#### 2.3.1. Mobile Application Interface

The mobile application had nine interfaces. The figures below show the interfaces of mobile applications known as the SpO2 analyzer.  Figure 11 shows the logo of the mobile application.

Figure 12 shows the login interface of the mobile application. Old users can login by using their username and password, and new users need to sign up to login.

Figure 13 shows the sign-up interface of the mobile application. New users can sign up to login by providing their usernames, email addresses, and passwords. After completing the sign up, the user's data will be stored in the cloud platform firebase, and after successfully signing up, the user can see a new interface with a login button. By clicking the login button, the user can login to the mobile application.

Figure 14 shows the user portal interface. After successfully logging in, this interface will appear. By clicking on the normal user button, the patient can check their measured data. Doctors can monitor their patients' measured data by clicking on the doctor portal. There is also a button named “Logout.” Users need to logout from the mobile application by clicking on the logout button.

Figure 15(a) shows the normal user interface. When the patient clicks on the normal user button, this interface will appear. In this interface, by clicking on the check health condition, the user can see the measured oxygen saturation and pulse rate data. When the user clicks on the tap to connect to the server button, the mobile application will connect to the device and show the measured SpO2, temperature, and pulse rate of the patient.  Figure 15(b) shows the measured SpO2, pulse rate, and temperature interface.

Figure 16(a) provides the doctor portal interface. When the doctor clicks on the doctor's portal button, this interface will appear. In this interface, doctors can analyze normal and COVID-19 patients' temperatures, SpO2, and pulse rates by clicking on the normal patient and COVID-19 patient buttons, respectively.  Figure 16(b) shows the normal patient portfolio. When the user clicks on the normal patient button, this interface will appear. If there is any normal patient who is not affected by COVID-19, then this interface will show the list of normal patients.

When the user clicks on the COVID-19 patient portfolio, this interface will appear as shown in Figure 17. By clicking on the check patient button, the doctor can see the patient's measured temperature, SpO2, and pulse rate, as shown in Figure 17.

## 3. Results

The system consists of two parts: the hardware and the mobile application. Both parts are essential for the system, and users can obtain results from both. This system was built by the circuit diagram and flow chart as shown in Figures 2 and 3.  Figure 18 shows the system prototype. Here, the Arduino Uno, LCD display, buzzer, pulse sensor, temperature sensor, node MCU, and Bluetooth module were added to implement the system. In the display of the system, the measured pulse rate, SpO2 level, and body temperature are shown; if the measured pulse rate and SpO2 level go out of range, the buzzer rings. This system prototype is simple and easy to use. It may be easily moved from one location to another because it is a lightweight prototype. Because all of the components are precisely positioned, the overall result is satisfactory.

After examining the system separately, it was observed that the system worked adequately. This means that the system design and implementation process for the project were correct; thus, the user's data were satisfactorily measured. The full system has two combined main parts. Through this system, users can obtain measured values of their vital signs through the mobile application as well as the LCD of the system.

The system was tested on a real human test subject.  Figure 19 shows the user experience and measured values of vital signs for the user. The LCD and mobile applications show the measured heart rate, SpO2, and temperature, in which the user can see the displayed results from the system. This system passes the data to a mobile application, which is one of its crucial parts. Through this device, users can obtain the required results through a mobile application; thus, this method is user-friendly and convenient. The system worked successfully.

Figure 20 shows the measured values of SpO2, pulse rate, and temperature of the user. It is an important interface for mobile applications because it provides the main results of the system. All sensors worked satisfactorily.

This device was used by five people aged between 23 and 56 years. It provided precise values for all features that have been included in this system.  Table 2 lists the measured values for the five users and the measured values of SpO2 level, pulse rate, and temperature. According to Table 2, the SpO2 level of most people is 97, which is close to the standard values. For the pulse rate, the measured values for the different subjects were comparable. The measured physiological data were different for different test subjects. All of these measured values were accurate compared to those of other commercially available devices. From Table 1, it is inferred that this system is reliable and user-friendly.

## 4. Conclusions

The COVID-19 pandemic has resulted in a global health crisis as thousands of people die from the disease every day. The fatality rate can be minimized if proper treatment is administered at the right time. Various steps, including regular monitoring of pulse rate, SpO2 level, and temperature, have been taken to ensure proper treatment. However, the oxygen level of a COVID-19 patient decreases with time, and the patient can die shortly if emergency steps are not taken. Considering the abovementioned facts, an IoT-based smart health monitoring system was developed for COVID-19 patients. The system runs through an IoT-based mobile application, and both the doctor and the patient can receive alerts from this system during emergencies. Therefore, individuals can use this system effectively anywhere. Advanced features can be added in the future because the entire system is IoT-based.

Moreover, this study broadly explores the components utilized within the system and the usefulness of each component. It provides a list of strategies that can be actualized to plan this system. From the beginning of the development of this system, we aimed to develop a well-organized application-based device that could be used in the current pandemic. COVID-19 patients and people enduring numerous other infections like chronic obstructive pulmonary disease (COPD) and asthma can use this gadget. The system is cost-effective, noninvasive, and versatile in nature, which makes it easier to screen patients' well-being regardless of where they are. Additionally, it provides real-time alerts to concerned individuals and medical experts about any circumstance that requires prompt consideration. This system can offer assistance to guarantee appropriate medical care all over Bangladesh, including in rural zones, thereby decreasing the number of patients. Early distinguishing proof of any medical condition can help the patient to take essential critical measures, which can possibly save the patient's life. Therefore, to make all lives risk-free, we must use smart health monitoring systems. To conclude, this system is extremely important in the medical sector because it can help increase the life expectancy of people worldwide. In the future, more sensors can be added to this system to monitor more physiological parameters of the human body.

## Figures and Tables

**Figure 1:** Block diagram of the system.

**Figure 2:** Flow chart of the system.

**Figure 3:** Block diagram of the circuit system.

**Figure 4:** Arduino Uno [25].

**Figure 5:** Pulse Sensor (MAX30100) [27].

**Figure 6:** Bluetooth module [29].

**Figure 7:** Node MCU ESP8266 [31].

**Figure 8:** Buck converter [32].

**Figure 9:** 16 × 2 LCD display.

**Figure 10:** DS18B20 Sensor [32].

**Figure 11:** Mobile application logo.

**Figure 12:** Login interface of mobile application.

**Figure 13:** (a) Sign up interface of mobile application and (b) successful sign up.

**Figure 14:** User's portal interface of mobile application.

**Figure 15:** (a) Normal user interface of mobile application. (b) Measured SpO2, pulse rate, and temperature.

**Figure 16:** (a) Doctor portal interface of mobile application. (b) Normal patient portfolio of mobile application.

**Figure 17:** Measured SpO2, pulse rate, and temperature.

**Figure 18:** Prototype of the system.

**Figure 19:** User experience (device is testing for real human test subject).

**Figure 20:** Measured value of user in mobile application.

**Table 1:** Lists of the required hardware components, their quantity, and cost of the products.

Item description	Unit price	Quantity	Total price (BDTK)
Arduino Uno	420	1	420
Temperature sensor	450	1	450
SpO2 Pulse Sensor	1400	1	1400
Node MCU Wireless Module	525	1	525
Bluetooth module	280	1	280
16 × 2 LCD display	285	1	285
Buck converter	82	1	82
3.7 lithium battery	60	2	120
3.7 lithium battery protector	45	2	90
2 s lithium battery	1850	1	1850
2 s lithium battery protector	250	1	250
9 V 2A battery adapter	100	1	100
Wire set	120	2	240
Switch	10	1	10
Buzzer	18	1	18
Total			6120

**Table 2:** TheSpO2, pulse rate, and temperature values of 5 different users from this system.

Person	Age	SpO2 (%)	Pulse (bpm)	Temperature (C)
Person 01	25	97	75	37
Person 02	32	97	73	36
Person 03	34	93	70	40
Person 04	56	97	74	37
Person 05	23	97	75	40

## Data Availability

No data was utilized to support these research findings.
